The article "Protein-Protein Interaction Analysis through Network Topology (Oral Cancer)" was published in 2021. Journal: J Healthc Eng.

# Protein-Protein Interaction Analysis through Network Topology (Oral Cancer)

**DOI:** 10.1155/2021/6623904

**Published:** 2021-01-16

**Authors:** Fazal Wahab Khattak, Yousef Salamah Alhwaiti, Amjad Ali, Mohammad Faisal, Muhammad Hameed Siddiqi

**Affiliations:** ^1^Department of Computer and Software Technology, University of Swat, Mingora, KPK, Pakistan; ^2^Department of Computer Science, Al Jouf University, Sakaka, Aljouf, Saudi Arabia; ^3^Department of CS & IT, University of Malakand, Chakdara, KPK, Pakistan

## Abstract

Oral cancer is a complex disorder. Its creation and spreading are due to the interaction of several proteins and genes in different biological thoroughfares. To study biological pathways, many high-yield methods have been used. Efforts to merge several data found at separate levels related to biological thoroughfares and interlinkage networks remain elusive. In our research work, we have proposed a technique known as protein-protein interaction network for analysis and exploring the genes involved in oral cancer disorders. The previous studies have not fully analyzed the proteins or genes involved in oral cancer. Our proposed technique is fully interactive and analyzes the data of oral cancer disorder more accurately and efficiently. The methods used here enabled us to observe the wide network consists of one mighty network comprising of 208 nodes 1572 edges which connect these nodes and various detached small networks. In our study, TP53 is a gene that occupied an important position in the network. TP53 has a 113-degree value and 0.03881821 BC value, indicating that TP53 is centrally localized in the network and is a significant bottleneck protein in the oral cancer protein-protein interaction network. These findings suggested that the pathogenesis of oral cancer variation was organized by means of an integrated PPI network, which is centered on TP53. Furthermore, our identification shows that TP53 is the key role-playing protein in the oral cancer network, and its significance in the cellular networks in the body is determined as well. As TP53 (tumor protein 53) is a vital player in the cell division process, the cells may not grow or divide disorderly; it fulfills the function of at least one of the gene groups in oral cancer. However, the latter progression in the area is any measure; the intention of developing these networks is to transfigure sketch of core disease development, prognosis, and treatment.

## 1. Introduction

Verbal cancer, mouth cancer, and head and neck cancer are all related to each other [1], which are cancers affecting cell development or found in the oral cavity [2]. They may occur as an essential injury beginning in any of the tissues within the oral cavity; its reason may be metastasis process occurring away from oral cavity or is due to change in neighbor physical structures, such as the nasal cavity. Or the oral cancers may originate in any of the mouth tissue and can spread to any cell or tissue: teratoma, adenocarcinoma inferred from a saliva gland, and tonsillar or other lymphoid tissues cause lymphoma; pigment-producing cells of the oral mucosa are producer of melanoma. Oral cancers are of few kinds, but almost 90% originate within the tissues that join the mouth and lips called squamous cell carcinomas [3].

Oral cancer is the most common cancer in the world with low overall survival rates [4], where oral squamous cell carcinoma (OSCC) is the most common type [5]. The organs that suffer from oral cancer include the buccal mucosa, tongue, and lower lip, and it mostly occurs in the people whose age is more than fifty years [6]. Traditional manual methods for creating network books, diagrams, or maps have been in use for a long time. The diagrams and other visual data in these valuables were handmade decades ago and have only restricted use. These graphs were based on information of that specific time when created, consisting of unchangeable and interaction less data.

Various biological procedures are enunciated as systems. Networks are demonstrated from the field of atomic sciences such as metabolic networks, protein interaction networks, and gene regulatory networks. Network analysis, sculpting, and visualization are imperative stride about a framework's natural perception of living beings. The visual interpretation of such networks gives the basic idea about the structure of network and also can create an idea about newly generated complex biological data [7].

Genetically, oral cancer has still not been fully analyzed and explored even after several years of research. Many casual or susceptible genes associated with oral cancer have been reported in the research studies. Thus, the focus of our research work is to obtain results that give us useful data related to genes involved in oral cancer and enable us to draw conclusions about gene-gene and related protein-protein interactions.

## 2. Literature Review

The role of proteins networks in syndromes identification and analyses is very significant. Throughout a period, study in miniature creatures and protein networks plays a vital role in molecular development study enhancement to increase vision in the strength of cells to disruption and also for allotment of new protein occupations. Succeeding those investigations and the present increase of protein interactivity capabilities in mammals, protein networks are progressively helping as toolkit to unknot the molecular foundation of disease. The authors of this paper review favorable uses of protein networks in disease in four main parts:

- Latest disease genes identification
- Study of their network valuables
- Spotting disease-linked subnetworks
- Network-based disease sorting

Proteins networks can also be used in areas like infectious disease, self-medication, and pharmacology [8].

Due to interaction detection methods, millions of interactions between proteins have been discovered. Focus of the paper is based on the graph theory, and the authors derived a new method from graph theory known as spectral method. Spectral method was used to disclose unseen networked structures of complex protein-protein collaboration networks. They come up with the idea that these concealed topological layouts comprise organically germane serviceable clusters. This idea stirs a novel approach to forecast the function of unknown proteins based on the classification of known proteins within network structures. With the use of this procedure, 48 quasi-cliques and six quasi-bipartite were separated from a network consisting of 11855 interactions among 2617 proteins in budding yeast, and 76 uncharacterized proteins were allocated functions [9].

All biological processes were considered important and specifically achieved through protein-protein interactions. They use spectral analysis method as a technique to disclose high-level structures using colossal and multifaceted associations. the structurae of the image radius that the authours obtained by the speculative analysis is used in the nalysis for the topology making is used in the analysis for the topology making for the disclosure of unseen topological structures of a complicated interface network [9].

Proteome functional organization can understand better by using human PPI for the identification of interrelating sets of human proteins scientifically; a protein matrix of 4456 baits and 5632 victims was separated by predetermined yeast two-hybrid (Y2H) interaction coupling. They acknowledged 3186 frequently original relations among 1705 proteins, which produce a huge, highly connected network, following Y2H technique. The Y2H scheme is an influential PPIs identification tool, applicable to high-throughput method in detection of complete proteome of organism interactions. To describe high-level confidence relation among proteins, different techniques were used, for example, topological, GO criteria and scoring system. The network was also used to locate genes without any character assigned to humans' disease proteins players in regulating the cellar trials. Screening human proteins relations systematically can enhance the understanding of protein functionality and cellular procedures [10]. They present their experiments results in the form of different graphs and charts.

There are a huge number of collaboration networks; studying them, finding functional nodes and links, and investigating the inner function of cells are the aims of this research. The authors performed a precise chart theory-based examination of this PPI arranged to build computational models for relating and anticipating the properties of deadly changes and proteins contributing in hereditary contacts, utilitarian bunches, protein complexes, and signaling pathways. Their examination suggests that deadly modifications are not as it were exceedingly related inside the organize structure, but they moreover fulfill an extra property. Their evacuation causes a diversion in organized structure. Creators moreover give proof for the nearness of diverse ways that maintain a strategic distance from practical proteins in PPI systems, whereas such ways do not exist for lethal change [11].

The PPI network includes a minor quantity of exceedingly associated protein hubs (also called centers) and various ineffectively associated hubs. Genome-wide consideration shows that cancellation of a center protein is more likely to be hazardous than cancellation of a nonhub protein; a wonder known as the centrality-lethality runs the show. This run of the show is commonly accumulated to reflect the unprecedented centrality of centers in organizing the courses of action of qualities, which in turn suggests the normal importance of organize plans, a key conviction of frameworks of science. Concurring to creators, for the notoriety of this clarification, the fundamental cause of the centrality-lethality running the show has never been basically inspected. They propose the concept of basic PPIs to discover out PPIs that are vital for the presence or propagation of a life form. As anticipated, basic PPIs are developmentally more moderated than insignificant PPIs. Considering the part of basic PPIs in deciding quality essentiality, they discover the yeast PPI organize practically more energetic than arbitrary systems, however with less distant sound than the potential ideal. These and other discoveries give unused viewpoints on the organic centrality of arranged structure and vigor [12].

Genomic consideration shows that erasing an exceedingly associated protein hub (center) is more likely to be deadly to a living being than erasing a humble associated hub (nonhub), a strategy recognized as the centrality-lethality running the show. As center points are more imperative than nonhubs in organizing the worldwide arranged structure, the centrality-lethality running the show is broadly accepted to reflect the worth of organized engineering in characterizing organized work, a key idea of frameworks science. Consequently, the centrality-lethality running the show is clarified without the association of organized engineering. Utilizing yeast information, the creators gave down to earth confirmation supporting their speculation [12].

In paper [13], ARIYA et al. suggested a microRNA consisting of multiple genes; actually microRNAs are analyzed, which seemed to be fruitful in high level of tumor. They veiled for the genetic factor; the appearance of these genetic factor remained associated with oral cancer development and evolution. Therefore, recognizing medications that might aim at these genetic factors might benefit plummeting the oral cancer humanity by cultivating development of patients.

In paper [14] by amiri et al., the scheme method has been planned to reconnoiter hereditary difficulty of oral cancer besides recognizing innovative oral cancer associated genes to perceive genomic modifications at molecular smooth, as concluded from variance investigation. Their genetic and communicating examination indicated important enhancement metabolism, motioning trail, and microRNA trails on the road to development. Their integrative method would benefit discovering the genetic variants of oral cancer that can speed up drug detection consequences to mature a healthier sympathetic concerning action approaches for numerous cancer categories.

Protein-protein interaction (PPI) network analysis of cancer has gained focus of medical and biological scientists. Through this approach, examination of the interaction between genes that cause cancer could lead us to improve the diagnosis and treatment of patients [15, 16]. In PPI network analysis, the genes related to the disease are gathered and organized in an integrative structure [15, 17]. The calculation of topological properties of the network, including central parameters such as degree and centrality, provides useful information about molecular mechanism of disease onset and pathology [18]. Introducing selected genes among large number of query genes can lead to specific biomarker panel related to the disease [19].

## 3. Methodology

The methodology of protein-protein interaction of oral cancer consists of seven steps. The first step is the attainment of the candidate genes of oral cancer, which was done in two ways: Firstly, PolySearch text-mining system is used, which is a web-based tool exploiting various techniques to highlight and align informative text. PolySearch results gave us a large list of genes and proteins. A lot of data are available on cancer. As our specific target is to collect and analyze data on oral cancer, PolySearch tool is used for obtaining the specific data on oral cancer. Secondly, we manually confirmed from reviewing the literature that the obtained genes and proteins were indeed of oral cancer. The second step of the methodology involved the use of STRING database for scanning the protein interactions. Construction of PPI networks, from which an extended network was derived, was used to extract the giant component making up the third step. The fourth step involved the analysis of the PPI network based on its topology. The fifth step was the creation of a backbone network from the giant network based on the highest betweenness centrality (BC) value. The sixth step involved the construction of a subnetwork from the giant network that consisted of all shortest routes among the aspirant genes. The seventh step concluded with TSPO as central protein.

### 3.1. Dataset Preparation for the Extraction of Genes Associated with Oral Cancer

Candidate genes associated with oral cancer were searched using PolySearch text-mining system, which is a useful tool in producing a list of ideas based on the query of the user. PudMed, OMIM, Drug Bank, and Swiss-Prot are among the few sources of information from which data relevant to the query can be extracted. PolySearch contributes a great deal to extracting information on important biomedical concepts such as genes/proteins, disease, SNPs, drugs, metabolites, pathways, and tissues, which could help in finding the relevant genes of oral cancer [20]. This method is used for finding genes related to oral cancer. Search was performed using the key words “Disease with Gene/Protein Association” and “Oral Cancer.” The literature analysis by PolySearch system returned 274 results. To determine the accuracy, these results were confirmed manually to check whether oral cancer associated genes were viable candidates or not. Discarding the less significant genes resulted in a total of 208 candidate genes for oral cancer by literature survey (Table 1).

### 3.2. Scanning Protein-Protein Interactions

Oral cancer candidate genes listed in Table 1 were converted to seed proteins. For visualizing the PPIs, STRING database was used. It is an exploratory database for PPIs. Updated version of STRING, 9.1, contains more than 1100 organisms, covering millions of proteins [20].

### 3.3. Constructing PPI Network from the Extension for Extraction of the Giant Component

A system, which consisted of the seed proteins and has also direct association with their PPI's neighbors, was developed. This system was built using Cytoscape [21], which is an extremely flexible project designed for the purpose of investigations, operations, and visualization of extensive systems. Not only did this study involve expansion on the system incorporating a giant part but also it included two small separate parts. The expectation of this study was that the giant network must consist of hubs with extensive BC value. This was clearly in light of the fact that both separate parts consist of a small number of hubs, and for this purpose the investigation and preparation involved only the giant network with its various parameters. The use of giant system obtained from the extended system was examined and analyzed by this method advantageously.

### 3.4. Protein Interaction Network Involving Topological Analysis

For accessing the hubs in the system, nodes properties such as betweenness centrality (BC), closeness centrality (CC), and degree (K) were noted and used, especially K and BC values. Quantity of adjacent joints which is based on the determination of the number of connections of one protein to its neighbors determines the most important factor, that is, the degree (K). The number of shortest routes that pass through each node, thus measuring the frequent occurrence of the node which has the greatest restricted routes between other nodes, determines the betweenness centrality. Shortest path or the most limited way is found by measuring the length of every last one of the geodesics to or from the network. The flow in the network is characterized by a high BC node value to great extent. BC may assume an integral part as a global property, since it is a valuable pointer to distinguish bottlenecks in a system. The converse of the normal length of the briefest paths among all the other nodes in the graph, which let us know the topological focus of the network, constitutes a closeness centrality (CC). Estimates of networks based on global topology include average degree, mean most brief path length, and distances utilized in the network.

  Average degree (<K>): mean of total degree values of nodes in a network
  Mean shortest path length (mspl): represents connecting average of the steps involved to every pair of nodes using their shortest path
  Diameter (D): longest paths among all shortest paths, characteristics of nodes, and measurements used to characterize the network were calculated by Cytoscape software in this paper

### 3.5. Creating Backbone Network by Searching High BC

This study involved observing the PPI supporting the oral cancer-related gene network.

Consequently, the proteins with high BC ought to have vigorously utilized crossing points as the backbone actually consisted of these proteins and their connections within the network. The critical point with high BC value was set at top 15 genes of the total number of nodes within the network [9, 10]. BC nodes with high values and their interlinkage were mined utilizing the giant network for creation of a backbone network. Furthermore, BC also served the purpose of measuring the nodes centrality in the network initially since according to the definition, BC values that are high consist of the shortest paths in the network passing through the nodes. These nodes with high BC value are among other nodes of the network function as bottleneck control interaction.

### 3.6. Construction of a Subnetwork among the Candidate Genes with the Shortest Paths

Some of the candidate genes in the network are not directly connected and that includes the giant network as well. For constructing a subnetwork, genes connected with least number of nodes, in link with oral cancer, are required. For this, each combination of candidate qualities and their most limited way was calculated. These ways were found using Cytoscape software, coming about within the subnetwork comprising all nodes in these ways.

### 3.7. Central Protein TP53 Validates the Backbone Network

Validation was essential for checking the healthiness of the backbone network. For this, test networks were developed as they were employing a little component of 208 genes as initial seeds. For this, once more Cytoscape computer program was utilized. BC value was determined in these test networks. Segments having nodes with top 15 BC in the test networks agreed with the nodes in the backbone network as per description in the fifth step to determine the accuracy of the backbone. Furthermore, the healthiness of backbone network of oral cancer proteins was determined by calculation of the frequency of the nodes having the largest BC value which gives the accuracy of the backbone nodes.

## 4. Results

In this research work, we have obtained protein-protein interaction network through applying various steps discussed in the Methodology section. Then, we have obtained the key nodes involved in protein-protein interaction network and perform the analysis for obtaining important protein or genes involved in oral cancer.

### 4.1. Network with Protein-Protein Interactions

A huge network with several collapsed smaller networks, respectively, found from the seed proteins TSPO and TP53, was also a part of the extended network (Figure 1). Giant network contained of 208 nodes connected with 1572 edges as illustrated in (Figure 2). The backbone network, however, comprised 322 edges linking 29 nodes (Figure 3). Another network consists of 25 nodes linking 87 edges (Figures 4 and 5). The further distinguishing feature is the presence of some very highly connected nodes, though they are very small in number, while others show fewer connections.

### 4.2. Analysis of the Key Nodes Involved in the PPI Network

Key nodes were viewed by using nodes having large degree or high betweenness centrality values, and the critical point was set as 10% of the total number of nodes for both the degree and BC in the network in this study. Among the total 208 nodes, those that had high BC were 59 in number, and 109 nodes had a large degree. 10 nodes had a large degree and high betweenness centrality (Table 2), nodes among the high BC, CC, and degree nodes (Table 3). To visualize the role of each protein in the oral cancer network, different colors and sizes were assigned to highlight them (Figure 2). TP53 is a protein with largest degree, TPSO is a protein with highest BC value, and EGFR is a protein with highest CC value. TP53 occupies central position in the network due to its high degree, BC, and CC value. Signaling pathways in the high betweenness centrality network and their cross-talks are obtained from the backbone networks. 1st backbone network consists of 29 nodes and 322 edges (Figure 3). Second major backbone network consists of 25 nodes and 87 edges (Figures 4 and 5). Analyzing the values of BC and CC shows that TP53 locates at the center of the backbone network with the highest BC value and the largest degree. TP53 has 29 neighbors: CCND1, SMAD2, TSPO, MTOR, ICAM1, VEGFA, STAT3, EGR1, TERT, MMP1, CCND2, MET, AKT1, KDR, TP53, RAF1, IL6, EGFR, PTGS2, PTPN11, FGF2, CDKN2A, TGFB1, BIRC5, CDKN1B, PROM1, SMAD4, CDH1, and CDK4. Details of other proteins in the backbone network were not included here.

## 5. Discussion

Genetically oral cancer has not been fully explored; even after several years of research it still remains unexplored. Many casual or susceptible genes associated with oral cancer have been reported. The multiple factors contributing to hepatocarcinogenesis include ecological, transmissible, sustaining, metabolic, and endocrine structures, which are involved specifically or indirectly in the development of oral cancer. The oral cancer pathogenesis indicates the involvement of several genes and can broadly be classified into four majors groups: regulatory genes involved in response to DNA damage, cell cycle control players, those intricate growth inhibition, apoptosis, and also the genesis involved in cell-cell collaboration and signal transduction. Analyzing the contribution of genes and proteins pertaining to oral cancer pathogenesis in addition to the involvement of other key proteins in the PPI networks by analyzing their topology was the goal of this study. The results obtained gave us useful data related to genes involved in oral cancer and enabled us to draw conclusions about gene-gene and related protein-protein interactions. It was observed that most of the seed proteins (208) connected to giant network in terms of oral cancer and their PPI neighbors. This giant oral cancer network consisted of 1572 edges. Backbone network topology, however, resulted in different small network topologies. As it is not possible to draw conclusion from the giant network, we further split down the backbone network into small subnetworks for obtaining clear results on oral cancer. The splitting of backbone network is performed according to properties of nodes, that is, BC, CC, and degree values. One backbone network consists of 29 nodes and 322 edges. Another subnetwork consists of 27 nodes 87 edges. There is one small subnetwork of 4 nodes and 5 edges. Other subnetworks also exist but they are very small. Literature was analyzed to find further techniques and methods supporting the importance of different genes in oral cancer. TP53 is a gene that occupied important position in the network. TP53 has degree value of 113 and BC value of 0.03881821. Literature was analyzed to find further techniques and methods supporting the importance of TP53 in cancer. In this regard, researchers have clarified TP53 changes in different types of cancers. Moreover, it has been discovered that TP53 reaction pathway is regularly flawed in human diseases and the recurrence of TP53 fluctuates greatly. In another study conducted by Ding and colleagues, polymorphisms were affiliated with this disorder. The study was focused around metainvestigation to better comprehend the relationship between polymorphism of Condon 72 and the tumor protein p53 (TP53) gene, which results in a missense transformation of arginine (R) to proline (p) and causes vulnerability to hepatocellular carcinoma [22, 23]. TSPO is another important gene in oral cancer network having highest BC value of 0.04809981 and degree value of 93. TP53 mutation sites with stalk cell-like gene appearance in addition to association with many cancers were also found in oral cancer with high mortality rate, although the exact sites are unknown as of yet. Moreover, direct sequencing methods are more helpful for reliable results. Form direct sequencing result, it was concluded that TP53 mutations, mainly the blistering mutations R249S and V157F, are linked with meager prognosis for patients with oral cancer. The stem cell-like acquirement of gene manifestation traits might be a contributing factor to the violent behavior of tumors with TP53 mutations having shorter survival rate as compared to wild-type TP53, according to literature survey [23–25].

## 6. Conclusion

The mainstay network shows clearly all the essentials genes of oral cancer, their associated regulatory pathways, and the interactions between them. This eventually brought us to the conclusion that TP53 is the protein with the highest degree, TSPO is the protein with largest BC, and EGFR is the protein with highest CC values, but TP53 obtained the important position in the network due to its degree, BC, and CC values, indicating that TP53 is centrally localized in the network and is a significant bottleneck protein in oral cancer protein-protein interaction network. These findings suggested that pathogenesis of oral cancer variation was organized by means of an integrated PPI network, which is centered on TP53. Furthermore, our identification of TP53 as the bottleneck protein in oral cancer network determined its significance in cellular network in the body as well, as P53.

Tumor protein 53 is important in the regulation of cell division; by restricting the cells from growing or dividing uncontrollably, it fulfills the function of at least one of the gene groups in oral cancer.

## Figures and Tables

**Figure 1:** Illustration of the extended network, which includes the huge network and some smaller networks. The labeled nodes are known as seed proteins, which were within the list of candidate genes, shown in Table 1.

**Figure 2:** Illustration of giant network topology. This huge network, which was derived from the extended network, is its biggest segment. BC values indicate the size of nodes.

**Figure 3:** Illustration of the backbone obtained from other networks. It consists of 29 nodes with highest betweenness centrality, and nodes' size indicates their BC values.

**Figure 4:** Illustration of the backbone obtained from other networks. It consists of 25 nodes and 87 edges.

**Figure 5:** Illustration of the backbone obtained from other networks. It consists of 4 nodes and 5 edges with highest betweenness centrality.

**Table 1:** List of genes showing association with oral cancer, extracted from the literary database.

SN	Symbol	SN	Symbol	SN	Symbol	SN	Symbol	SN	Symbol	SN	Symbol	SN	Symbol	SN	Symbol	SN	Symbol	SN	Symbol	SN	Symbol
1	ABCA1	20	CASP7	39	CP	58	DSC2	77	GPX1	96	IL6	115	MT1A	134	PHLDA1	153	REST	172	SMC2	191	TNFSF10
2	ABCE1	21	CCL20	40	CSNK1E	59	DSG1	78	GRIK2	97	ITGB2	116	MT3	135	PIK3CA	154	RPL30	173	SMURF1	192	TP53
3	ADAM17	22	CCL5	41	CXCL2	60	DSG2	79	GRM5	98	ITGB4	117	MTA1	136	PIM1	155	RPL37A	174	SOD2	193	TP73
4	AKT1	23	CCND1	42	CXCL3	61	DUSP1	80	GSK3A	99	KDR	118	MTHFR	137	POFUT1	156	RPS17	175	SOX2	194	TSPO
5	ALCAM	24	CCND2	43	CXCR1	62	E2F1	81	GSTM1	100	KLF4	119	MTOR	138	POLG2	157	S100A1	176	SRF	195	TWIST1
6	ANG	25	CCNH	44	CXCR2	63	EDNRB	82	GSTO1	101	KLF8	120	MVD	139	POLRMT	158	S100A2	177	ST14	196	TXNRD2
7	ANKRD6	26	CCR4	45	CXCR7	64	EGFR	83	GSTP1	102	KRT19	121	MYCBP	140	PRDM14	159	S100A4	178	STAG2	197	UBB
8	ANXA1	27	CD14	46	CYP1A1	65	EGR1	84	HBA1	103	LAMC2	122	NAT2	141	PREX2	160	S100A7	179	STAT3	198	VEGFA
9	APC2	28	CD207	47	CYP26B1	66	ELAVL3	85	HMGA2	104	LBX1	123	NES	142	PRKAB1	161	S100A9	180	TERT	199	WIF1
10	ATP2A2	29	CD44	48	CYP2E1	67	ENG	86	HMGB1	105	LCN2	124	NNMT	143	PROM1	162	S100B	181	TFRC	200	WNT2B
11	ATP2A3	30	CD68	49	DCN	68	ERCC2	87	HNRNPD	106	LDHA	125	NRP1	144	PROX1	163	S100P	182	TGFB1	201	WWP1
12	AURKA	31	CDH1	50	DCTN6	69	FADD	88	HOXA10	107	LIN28B	126	OAZ1	145	PTGS2	164	SEMA3C	183	TGFBR1	202	XRCC1
13	AXIN2	32	CDK4	51	DDX3X	70	FAM48A	89	HOXA9	108	MAPK14	127	OPRM1	146	PTMA	165	SF3B3	184	TGFBR2	203	XRCC2
14	BECN1	33	CDKN1B	52	DIABLO	71	FGF2	90	HPSE	109	MET	128	ORAOVA1	147	PTPN11	166	SIRT1	185	TIMP3	204	XRCC3
15	BIRC5	34	CDKN1C	53	DICER1	72	FHIT	91	HSPA5	110	MGMT	129	PABPN1	148	PTPRJ	167	SIRT3	186	TIMP4	205	XRCC4
16	BNIP2	35	CDKN2A	54	DNAH8	73	GAD1	92	HSPG2	111	MMP1	130	PARP1	149	PTPRR	168	SLC2A1	187	TLR2	206	YES1
17	BRCA2	36	CHAF1A	55	DNAJA3	74	GDNF	93	ICAM1	112	MMP7	131	PDK1	150	PTPRZ1	169	SLPI	188	TLR3	207	ZBTB7A
18	CA9	37	CHAF1B	56	DNMT3B	75	GHRL	94	ICAM3	113	MOK	132	PDPN	151	RAF1	170	SMAD2	189	TLR4	208	VEGF
19	CALML3	38	COL17A1	57	DPAGT1	76	GJA1	95	IL1F10	114	MSI1	133	PGK1	152	RASGRP3	171	SMAD4	190	TNFRSF11B		

**Table 2:** List of the proteins having high BC and large degree values.

SN	Gene	Degree	BC
1	TSPO	93	0.04809981
2	TP53	113	0.03881821
3	AKT1	90	0.01744922
4	EGFR	79	0.01611723
5	VEGFA	60	0.01249361
6	IL6	60	0.00829916
7	MTOR	49	0.00784171
8	CDH1	66	0.00782314
9	CXCR2	17	0.00712798
10	SMAD4	39	0.00692481

**Table 3:** Nodes with high BC, CC, and degree values.

Gene	Degree	Gene	CC	Gene	BC
TP53	113	EGFR	0.75409836	TSPO	0.04809981
TSPO	93	MAPK14	0.75	TP53	0.03881821
AKT1	90	CDKN1B	0.75	AKT1	0.01744922
EGFR	79	CDK4	0.73684211	EGFR	0.01611723
CDH1	66	TSPO	0.69767442	VEGFA	0.01249361
CCND1	61	STAT3	0.6875	IL6	0.00829916
VEGFA	60	IL6	0.67741935	MTOR	0.00784171
IL6	60	CD68	0.66666667	CDH1	0.00782314
STAT3	56	CHAF1A	0.66666667	CXCR2	0.00712798
FGF2	53	OAZ1	0.66666667	SMAD4	0.00692481
MTOR	49	EGR1	0.64705882	XRCC3	0.00531283
MAPK14	49	FGF2	0.63829787	MET	0.00516178
CDKN2A	47	BIRC5	0.63513514	UBB	0.00501709
TGFB1	47	MMP1	0.63218391	PARP1	0.00451757
KDR	42	RAF1	0.63157895	GJA1	0.00447296

## Data Availability

The data used to support the findings of this study are included within the article.
